# Mesenchymal stem cell-derived exosomes exert ameliorative effects in type 2 diabetes by improving hepatic glucose and lipid metabolism via enhancing autophagy

**DOI:** 10.1186/s13287-020-01731-6

**Published:** 2020-06-08

**Authors:** Qin He, Lingshu Wang, Ruxing Zhao, Fei Yan, Sha Sha, Chen Cui, Jia Song, Huiqing Hu, Xinghong Guo, Mengmeng Yang, Yixin Cui, Yujing Sun, Zheng Sun, Fuqiang Liu, Ming Dong, Xinguo Hou, Li Chen

**Affiliations:** 1 Department of Endocrinology, Qilu Hospital of Shandong University, No. 107 Wenhua Xi Road, Jinan, 250012 Shandong China; 2 Institute of Endocrine and Metabolic Diseases of Shandong University, Jinan, 250012 Shandong China; 3 Key Laboratory of Endocrine and Metabolic Diseases, Shandong Province Medicine & Health, Jinan, 250012 Shandong China

**Keywords:** Exosome, Mesenchymal stem cell, Glucose metabolism, Type 2 diabetes mellitus, Autophagy

## Abstract

**Background:**

Mesenchymal stem cell (MSC)-based therapy is currently considered to be an effective treatment strategy for diabetes and hepatic disorders, such as liver cirrhosis and non-alcoholic fatty liver disease. Exosomes are important mediators of cellular connections, and increasing evidence has suggested that exosomes derived from MSCs may be used as direct therapeutic agents; their mechanisms of action, however, remain largely unclear. Here, we evaluated the efficacy and molecular mechanisms of human umbilical cord MSC-derived exosomes (HucMDEs) on hepatic glucose and lipid metabolism in type 2 diabetes mellitus (T2DM).

**Methods:**

HucMDEs were used to treat T2DM rats, as well as palmitic acid (PA)-treated L-O2 cells, in order to determine the effects of HucMDEs on hepatic glucose and lipid metabolism. To evaluate the changes in autophagy and potential signaling pathways, autophagy-related proteins (BECN1, microtubule-associated protein 1 light chain 3 beta [MAP 1LC3B]), autophagy-related genes (ATGs, ATG5, and ATG7), AMP-activated protein kinase (AMPK), and phosphorylated AMPK (p-AMPK) were assessed by Western blotting.

**Results:**

HucMDEs promoted hepatic glycolysis, glycogen storage, and lipolysis, and reduced gluconeogenesis. Additionally, autophagy potentially contributed to the effects of HucMDE treatment. Transmission electron microscopy revealed an increased formation of autophagosomes in HucMDE-treated groups, and the autophagy marker proteins, BECN1 and MAP 1LC3B, were also increased. Moreover, autophagy inhibitor 3-methyladenine significantly reduced the effects of HucMDEs on glucose and lipid metabolism in T2DM rats. Based on its phosphorylation status, we found that the AMPK signaling pathway was activated and induced autophagy in T2DM rats and PA-treated L-O2 cells. Meanwhile, the transfection of AMPK siRNA or application of the AMPK inhibitor, Comp C, weakened the therapeutic effects of HucMDEs on glucose and lipid metabolism.

**Conclusions:**

These findings demonstrate that HucMDEs improved hepatic glucose and lipid metabolism in T2DM rats by activating autophagy via the AMPK pathway, which provides novel evidence suggesting the potential for HucMDEs in clinically treating T2DM patients.

## Background

Glucose metabolism in the liver plays a key role in maintaining stable blood glucose concentrations [1]. In patients with type 2 diabetes mellitus (T2DM), glucagon is inappropriately increased due to a loss of insulin inhibition, leading to increased liver glycogen decomposition and hyperglycemia [2]. In addition, elevated serum lipids are risk factors that cause atherosclerosis and progress diabetes [3]. Therefore, improving liver glucose and lipid metabolism represents an important strategy in the treatment of diabetes.

Cell-based therapy has emerged as a promising treatment strategy for diabetes [4]. Mesenchymal stem cells (MSCs) can be isolated from various tissues—such as bone marrow, mobilized peripheral blood, umbilical cord, and adipose tissue—and have played increasingly important roles in regenerative medicine [5, 6]. Human umbilical cord-derived MSCs (HucMSCs) have higher proliferative potential and lower immunogenicity compared with those of other MSCs and have become an ideal choice in treating diabetes [7–9]. Increasing evidence has shown that MSCs exert therapeutic effects mainly through paracrine signaling [10]. As an important manifestation of paracrine signaling, exosomes have been considered to represent a promising cell-free therapy due to their multiple bioactivities and intercellular communication functions [11, 12]. Previous studies have demonstrated that HucMSC-derived exosomes (HucMDEs) exhibit similar therapeutic effects to those of HucMSCs and circumvent imperfections in HucMSCs [13]. Moreover, exosomes are also easier to quantify and maintain bioactivities during storage and transportation [13]. However, the therapeutic effects and molecular mechanisms of HucMSCs on liver glucose and lipid metabolism disorders in T2DM still remain largely unknown.

Autophagy is a cellular process that removes dysfunctional or damaged organelles through lysosomal degradation and recycles their products for cellular metabolic needs and is tightly controlled by a group of factors, including autophagy-related genes (ATGs), microtubule-associated protein 1 light chain 3 beta (MAP 1LC3), and BECN1 [14]. Previous studies have implicated that autophagy disorders are present in the pathogenesis of various human diseases such as cancer, infection, and metabolic disorders [15]. Singh et al. demonstrated that autophagy may help to remove excess lipid droplets in hepatocytes [16]. Harrell et al. confirmed that MSC-derived extracellular vesicles could activate autophagy and inhibit apoptosis in injured hepatocytes [12]. However, whether HucMDEs affect liver glucose and lipid metabolism in T2DM by inducing autophagy remains unknown.

In the present study, we established a T2DM model in rats using a high-fat diet (HFD) in combination with streptozotocin (STZ) and also established an insulin resistance model in L-O2 cells induced by 0.25 mM of palmitic acid (PA) for 48 h. We then evaluated the effects of HucMDEs on hepatic glucose and lipid metabolism in vivo and in vitro. Finally, we demonstrated a correlation between HucMDEs, hepatic glucose/lipid metabolism, and autophagy, and further explored the potential mechanisms underlying this association. Taken together, our results provide novel ideas and a scientific basis for HucMDE intervention strategies in T2DM and related liver dysfunction.

## Methods

### Cell culture and treatments

With the approval of the Ethics Committee at Qilu Hospital of Shandong University, we obtained fresh human umbilical cords from full-term births by cesarean section. All participants provided informed consent for the use of the umbilical cord in this experimental study. The arteries and veins were removed after three washes in normal saline, after which the mesenchymal tissue, Wharton’s jelly, was exposed. Then, this tissue was cut into small pieces with sterile scissors, and these pieces were then placed in a cell culture bottle with α-MEM medium (Gibco, MD, USA) containing 20% fetal bovine serum (FBS, depletion of exosomes by ultracentrifugation; Gibco), within a 37 °C incubator with 5% CO_2_. We changed the culture medium every 3 days. The third to the seventh passage of cells were used for the experiments.

Human embryo lung fibroblast (HELF) and human L-O2 cells were purchased from the China Cell Culture Center (Shanghai, China) and were maintained in Dulbecco’s modified Eagle’s medium (DMEM, Hyclone, UT, USA) with 10% FBS, within a 37 °C incubator with 5% CO_2_. L-O2 cells were incubated with 0.25 mM of palmitic acid (PA, Sigma-Aldrich, USA) for 48 h to establish an insulin resistance cellular model [17]. L-O2 cells were pre-treated with HELF-derived exosomes (HDEs, 30 μg/ml, normal control exosomes) or HucMDEs (30 μg/ml) prior to PA treatment. To further evaluate the effect of HucMDEs on PA-induced changes in glucose and lipid metabolism, cells were pre-treated with autophagy inhibitor 3-methyladenine (3-MA, 10 mM, Sigma-Aldrich, USA), bafilomycin A1 (Baf, 20 nM, Sigma-Aldrich, USA), siATG5, siATG7, siAMPK, or an AMPK inhibitor (Comp C; 20 μM, Sigma-Aldrich, USA) before being cultured for 48 h in normal or PA medium.

### Animal experiments

Forty-two male 4-week-old Sprague-Dawley rats (~ 60 g each) were purchased from Synergy Pharmaceutical Bioengineering Co., Ltd. (Nanjing, China). After 2 weeks of adaptive feeding, rats were randomly divided into the following two groups: normal chow diet (control, *n* = 7) and 45% high-fat diet (HFD, *n* = 35). Four weeks after HFD feeding, these rats were then injected intraperitoneally with STZ (30 mg/kg, S0130; Sigma-Aldrich) after fasting for 12 h. The T2DM model was considered successful if there were two consecutive fasting glucose levels ≥ 16.7 mmol/l. T2DM rats were divided into five groups (*n* = 7/group): PBS, HELF, HucMSC, HDEs, and HucMDEs groups. Then, 5 × 10^6^ cells/rat of HELFs and HucMSCs in 200 μl of PBS were injected via the tail vein every week for 8 cycles after STZ injections as described previously [18]. HDEs and HucMDEs in 200 μl of PBS (10 mg/kg BW, which was the maximum tolerated dose [19]) were also injected via the tail vein every 3 days for 2 months, as previously described with minor modification [19–22] (see Supplementary Fig. 2 for more detailed experiment procedure).

In exosome-tracking experiments, HucMDEs (10 mg/kg of body weight [BW] in 200 μl of PBS) were labeled with Cy7 NHS ester (A8109, APExBIO, USA) and were delivered into T2DM rats via tail injection. The control group was infused with 200 μl of PBS. Perfused organs from fasted rats were imaged using an IVIS200 imaging system (Xenogen Corp., Alameda, CA, USA) at 24 h after harvesting the organs. During the experiment, no rats became severely ill or died. All animal experimental protocols were approved by the Animal Ethics Committee of Shandong University.

### Analysis of metabolic parameters

BW and fasting glucose were monitored weekly. Serum alanine aminotransferase (ALT), aspartate aminotransferase (AST), triglyceride (TG), and total cholesterol (TC) were detected after interventions via ELISA Kits (ColorfulGene Biological Technology, Wuhan, China). The intraperitoneal glucose tolerance test (IPGTT) was performed by the injection of glucose (1.5 g/kg, Sigma-Aldrich) after rats were fasted for 12–16 h. The intraperitoneal insulin tolerance test (IPITT) was performed by the injection of insulin (2 IU/kg, Wanbang Pharmaceutical, Jiangsu, China) after a 6-h fast. The blood was then collected from the tip of the tail vein at 0, 30, 60, 90, 120, and 180 min for glucose measurements.

### Isolation and identification of exosomes

For the isolation of exosomes, HucMSC-conditioned medium was collected and centrifuged at 300×*g* for 10 min to remove cells, followed by 2000×*g* for 20 min to remove cellular debris. The medium was centrifuged at 16,500×*g* for 30 min to remove microvesicles and was then filtered through a 0.22-μm filter. Finally, the medium was centrifuged at 120,000×*g* for 70 min at 4 °C. Exosomes were collected from the bottom of the tube and were either resuspended in PBS or lysed in RNA lysis buffer for further analysis.

Morphologies of exosomes were assessed via transmission electron microscopy (TEM; EM902A, Carl Zeiss MicroImaging GmbH, Germany). The sizes and relative intensities of exosomes were quantified by NanoSight NS300 (Malvern Instruments Ltd., UK). The expressions of CD9 and CD81 were detected by Western blotting.

### Exosomal tracing in L-O2 cells

HucMDEs were labeled using the PKH67 Green Fluorescent Cell Linker Kit (PKH67, Sigma-Aldrich) and were then incubated with L-O2 cells for 24 h. Cytoskeletons were visualized using rhodamine phalloidin (Cytoskeleton, Denver, MA, USA). Fluorescent signals were detected via confocal laser scanning microscopy TCS SP8 (Leica, Germany).

### Transmission electron microscopy

Liver tissues and L-O2 cells were prepared and subjected to TEM, as previously described [23]. Electron photomicrographs were taken of ultrastructures of liver tissues and L-O2 cells via TEM (JEM-1200EX II, JEOL; Tokyo, Japan).

### Western blot analysis

Cells or exosomes were harvested and lysed in RIPA buffer. Protein concentrations were detected with a BCA assay kit (P0012S, Beyotime, Shanghai, China). Transferred membranes were incubated overnight at 4 °C with the following primary antibodies from Cell Signaling Technology: MAP 1LC3B (2775), BECN1 (3495), ATG5 (2630), ATG7 (2631), AMP-activated protein kinase (AMPK, 5831), phosphorylated-(p-)AMPK (Thr172, 2535), and β-actin (3700). Additional antibodies that were used were as follows: GCK (Abcam, ab155962), PFK (Abcam, ab204131), PK (Abcam, ab171744), p-GSK3β (Abcam, ab68476), GSK3β (Abcam, ab62368), G-6-P (Abcam, ab167394), PEPCK (Abcam, ab133603), PPARα (Abcam, ab8934), and SREBP-1c (Proteintech, 14088-1-AP). After incubation with horseradish peroxidase-labeled secondary antibodies, protein bands were exported by the Image Lab software (BioRad, USA). Protein band intensities were measured via ImageJ and were normalized to β-actin.

### Small interfering RNA transfections

For RNA silencing, the sequences of small interfering RNAs (siRNAs) targeting human ATG5, ATG7, BECN1, and AMPKα were designed and synthesized by GenePharma (Shanghai, China). The sense and antisense sequences of ATG5 siRNA were 5′-CCT TTG GCC TAA GAA GAA A-3′. The sense and antisense sequences of ATG7 siRNA were 5′-GGA GTC ACA GCT CTT CCT T-3′. The sense and antisense sequences of BECN1 siRNA were 5′-GGA AGC TCA GTA TCAGAGA-3′. The sense and antisense sequences of AMPKα siRNA were 5′-GAGGAGAGC TAT TTG ATT A-3′. The normal control (NC) siRNA targeted the following sequence: 5′-UUCUCCGAACGUGUCACGUTT-3′. L-O2 cells were transfected with 160 pmol of siRNA for 6–8 h via Lipofectamine 2000 transfection reagent (Invitrogen, USA), according to the manufacturer’s instructions.

### Lentiviral transfections

GFP-MAP 1LC3B (pBABEpuro, 22405)-expressing vectors were purchased from Addgene (Cambridge, MA, USA). The constructs, transfections, and lentiviral infections of GFP-MAP 1LC3B that we used have been described previously [24]. After treatments, we calculated the number of autophagic cells expressed as GFP-MAP 1LC3B dots (positive cells as ≥ 3 dots). Images were scanned with an Olympus BX53 fluorescent microscope.

### Glycogen periodic acid Schiff staining

Periodic acid Schiff (PAS) staining was performed as previously described [25]. Liver sections and L-O2 cells were washed three times with PBS for 5 min and were then incubated with periodic acid for 8 min. After two washes in distilled water, the sections and cells were stained with Schiff reagent for 20 min, rinsed three times with distilled water, and were dyed with hematoxylin before microscopic examination.

### Statistical analyses

All experiments were repeated at least three times, and the results are reported as the mean ± standard deviation (SD). Statistically significant differences between the groups were determined by paired Student’s *t* tests or one-way analyses of variance (ANOVA) via the GraphPad Prism 7 software (San Diego, CA, USA). *P* < 0.05 was considered significant.

## Results

### HucMDEs improve glucose tolerance and increase insulin sensitivity in T2DM rats

Our previous study showed that MSCs could ameliorate oxidative stress-induced islet endothelium apoptosis and functional impairment in T2DM rats [18]. In order to determine whether MSC-derived exosomes exert similar therapeutic effects as those of MSCs in T2DM rats, HucMSCs and HucMDEs were first isolated and characterized. To begin identifying HucMSCs, surface markers and multilineage differentiation abilities of adherent cells were first examined. The results of oil red O staining and alizarin red staining showed that HucMSCs had the potential to differentiate into adipocytes (Fig. S1a) and osteoblasts (Fig. S1b). HucMSCs were then characterized using flow cytometric analysis to determine the presence of established surface markers of HucMSCs, such as CD105 and CD73. These markers were enriched in HucMSCs, while the negative markers, HLA-DR and CD34, had low expression (Fig. S1c).

HucMDEs were isolated and purified from HucMSC-conditioned media through standard exosome isolation via ultracentrifugation. Cup-shaped vesicles with a diameter of approximately 120 nm were identified by TEM (Fig. 1a) and NanoSight analysis (Fig. 1b). The exosomal protein markers, CD81 and CD9, were enriched in exosomes, while calnexin, an endoplasmic reticulum marker, was present in cells but absent in exosomes (Fig. 1c). PBS-treated and Cy7-labeled HucMDEs were subsequently injected via the tail vein. To assess the bio-distribution of HucMDEs, an in vivo imaging system (IVIS) was used to image live rats at 24 h after exosome injection (Fig. 1d). We found that HucMDEs were distributed in all harvested organs, including the heart, lung, liver, pancreas, spleen, kidney, and gastrointestinal tract (Fig. 1e).

**Fig. 1:** HucMDEs improve glucose tolerance and increase insulin sensitivity in T2DM rats. **a** TEM images of exosomes (scale bar 100 nm). **b** Particle sizes and concentrations of exosomes were measured by NanoSight analysis. **c** Western blotting showing characteristics of exosomes using the exosomal markers, CD81 and CD9, and the endoplasmic reticulum marker, calnexin. **d** IVIS showing the bio-distribution of HucMDEs in T2DM rats (left: PBS-treated control; right: Cy7-labeled HucMDEs) after 24 h of infusion. **e** Representative IVIS images of organs (heart, lung, liver, pancreas, spleen, kidney, and gastrointestinal tract) from rats (left: PBS-treated control; right: Cy7-labeled HucMDEs) after 24 h of infusion. **f** HELFs (5 × 10^6^ cells/rat, once every week), HucMSCs (5 × 10^6^ cells/rat, once every week), HDEs (10 mg/kg, once every 3 days), and HucMDEs (10 mg/kg, once every 3 days) in 200 μl of PBS were infused into T2DM rats. Fasting blood glucose was monitored once a week throughout the experiments. **g** Body weights of the following groups: Control + PBS, T2DM + PBS, T2DM + HDEs, and T2DM + HucMDEs. IPGTT and corresponding areas under the curve (**h**, **i**) and IPITT and corresponding areas under the curve (**j**, **k**) were performed to assess insulin tolerance and insulin sensitivity at 2 weeks after the last infusion of PBS, HDEs, or HucMDEs. All the results are expressed as the mean ± SD (*n* = 7 rats per group; *P < 0:05; **P < 0:01; ***P < 0.001)

We next established a T2DM rat model by HFD feeding followed by STZ injections. HucMSCs (5 × 10^6^ cells/rat, once every week) and HucMDEs (10 mg/kg, once every 3 days) were injected into T2DM rats via the tail vein, while HELFs (5 × 10^6^ cells/rat, once every week) and HDEs (10 mg/kg, once every 3 days) were injected as controls (Fig. S2). As shown in Fig. 1f, fasting blood glucose was significantly elevated after STZ injection and presented a dramatic fall after HucMDEs (10.64 ± 0.48 mmol/l) and HucMSC infusion (10.07 ± 0.29 mmol/l) (Fig. 1f), while PBS-, HELF-, and HDE-treated T2DM rats remained persistently hyperglycemic (19.66 ± 0.51 mmol/l vs. 18.02 ± 0.72 mmol/l vs. 17.97 ± 0.64 mmol/l, respectively). Meanwhile, HucMDEs significantly decreased weight loss in T2DM rats (Fig. 1g). The results of IPGTT (Fig. 1h, i) and IPITT (Fig. 1j, k) revealed that HucMDEs significantly ameliorated glucose metabolism and improved insulin sensitivity in T2DM rats. These data suggest that HucMDEs improved glucose tolerance and increased insulin sensitivity in T2DM rats.

### HucMDEs relieve liver dysfunction and improve lipid profiles in T2DM rats

We then verified the effects of HucMDEs on liver dysfunction and lipid profiles. Liver enzymes (ALT and AST) and serum lipid profiles (TC and TG) were markedly increased in T2DM rats compared with those in the control group and were decreased dramatically in HucMDE-treated T2DM rats compared with those in the HDE-treated group (Table 1), indicating that HucMDEs relieved liver dysfunction and improved lipid profiles in T2DM rats.

**Table 1:** HucMDEs relieve liver dysfunction and improve lipid profile in T2DM rats

	Control + PBS	T2DM + PBS	T2DM + HDEs	T2DM + HucMDEs
ALT (IU/l)	66.26 ± 5.10	100.62 ± 6.13**	103.71 ± 7.16	82.13 ± 6.13^#^
AST (IU/l)	195.23 ± 12.05	332.51 ± 16.58***	340.72 ± 18.45	293.05 ± 11.25^#^
TC (mmol/l)	1.95 ± 0.08	2.94 ± 0.14***	2.88 ± 0.15	2.16 ± 0.11^##^
TG (mmol/l)	0.78 ± 0.06	1.54 ± 0.08***	1.63 ± 0.10	1.23 ± 0.09^#^

After STZ induction and HDEs, HucMDE treatment for another 2 months, rats were anesthetized with chloral hydrate. Blood was collected to measure the levels of liver function (*ALT* alanine aminotransferase, *AST* aspartate aminotransferase) and the levels of lipid (*TC* total cholesterol, *TG* triglyceride). Data were presented as mean ± SD (*n* = 7). *P < 0:05; **P < 0:01; ***P < 0.001 (compared with the control group), ^#^*P* < 0:05; ^##^*P* < 0:01; ^###^*P* < 0.001 (compared with the T2DM + HDEs group)

### HucMDEs improve glucose and lipid metabolism both in vivo and in vitro

The liver plays a vital role in maintaining blood glucose balance by regulating glucose storage, production, and consumption. To evaluate the effects of HucMDEs in regulating glucose metabolism in vivo and in vitro, we employed a T2DM rat model and a PA-induced insulin resistance model in L-O2 cells. Then, PBS-treated and PKH67-labeled HucMDEs were co-cultured with L-O2 cells, after which cytoskeletons were visualized using incubation in rhodamine phalloidin for 24 h to detect exosomal uptake in L-O2 cells (Fig. S1d). Our results showed that glycolytic enzymes (GCK, PFK, and PK) and glycogen synthesis-related proteins (p-GSK3β/GSK3β) were decreased, while hepatic gluconeogenic enzymes (G-6-P and PEPCK) were increased in T2DM rats and PA-treated L-O2 cells compared to their corresponding control groups (Fig. 2a–c, f–h). PAS staining also showed a decrease in glycogen accumulation in T2DM rats and PA-treated L-O2 cells (Fig. 2d, i). HucMDE-treated T2DM rats and L-O2 cells had higher expression levels of glycolytic enzymes and p-GSK3β/GSK3β, whereas hepatic gluconeogenic enzymes were decreased compared with those in the T2DM and PA-treated groups (Fig. 2a–c, f–h). HucMDEs also increased PAS-positive staining in the livers and L-O2 cells in the model groups (Fig. 2d, i). The expression level of SREBP-1c, a transcription factor responsible for fatty acid synthesis, was increased in the livers of T2DM rats and in PA-treated L-O2 cells and was decreased after HucMDE intervention (Fig. 2e, j). PPARα, a nuclear receptor that participates in maintaining lipid homeostasis by regulating a series of target genes, was downregulated in the livers of T2DM rats and in PA-treated L-O2 cells and was upregulated in the HucMDE-treated group (Fig. 2e, j). Collectively, these data demonstrate that treatment with HucMDEs improved glucose and lipid metabolism both in vivo and in vitro.

**Fig. 2:** HucMDEs improve glucose and lipid metabolism both in vivo and in vitro. Glycolysis-related proteins (GCK, PFK, and PK) (**a**), glycogen synthesis-related proteins (p-GSK3β, GSK3β) (**b**), and gluconeogenesis-related proteins (G-6-P, PEPCK) (**c**) in the livers of the indicated groups were detected by Western blotting. **d** PAS staining in the livers of the indicated groups. **e** The hepatic lipid synthesis protein, SREBP-1c, and lipolytic protein, PPARα, in the livers of the indicated groups were detected by Western blotting. Glycolysis-related proteins (GCK, PFK, PK) (**f**), glycogen synthesis-related proteins (p-GSK3β, GSK3β) (**g**), and gluconeogenesis-related proteins (G-6-P, PEPCK) (**h**) in L-O2 cell groups of Control + PBS, 0.25 mM PA + PBS, PA + HDEs (30 μg/ml), and PA + HucMDEs (30 μg/ml) were detected by Western blotting. **i** PAS staining in L-O2 cells. **j** The hepatic lipid synthesis protein, SREBP-1c, and lipolytic protein, PPARα, in L-O2 cells of the indicated groups were detected by Western blotting. All the results are expressed as the mean ± SD (*P < 0:05; **P < 0:01; ***P < 0.001)

### HucMDEs induce autophagy in the livers and L-O2 cells

Growing evidence indicates that autophagy is widely involved in cellular metabolic regulation [26]. In addition, our previous studies have demonstrated that autophagy in chronic HFD-fed mice is dysregulated [23, 27]. Therefore, we next investigated autophagy levels in the livers of T2DM rats and in PA-induced L-O2 cells, as well as determined the effect of HucMDEs on autophagic flux. Downregulation of BECN1 and MAP 1LC3B-II, two markers of autophagy, occurred in the livers of T2DM rats and in PA-treated L-O2 cells compared to their corresponding control groups, while the expression of BECN1 and MAP 1LC3B-II recovered after HucMDE treatment (Fig. 3a, f). Moreover, HucMDEs markedly increased the percentage of GFP-MAP 1LC3B-positive L-O2 cells (Fig. 3b, c). TEM was then performed to detect autophagic vesicles, and the results demonstrated an increased production of autophagosomes (black arrows) in L-O2 cells (Fig. 3d, e) after HucMDE treatment. These results preliminarily indicated that HucMDEs induced autophagy.

**Fig. 3:** HucMDEs promote autophagy in the livers and L-O2 cells. **a** BECN1 and MAP 1LC3B protein expression levels in the livers of the indicated groups were analyzed by Western blotting. **b** L-O2 cells were transfected with Lenti-GFP-MAP 1LC3 and treated with PA (0.25 mM), HDEs (30 μg/ml), or HucMDEs (30 μg/ml) for 48 h (scale bar: 50 μm). **c** Percentages of cells with more than four GFP-LC3B dots were quantified. **d** TEM images showing the formation of autophagosomes (the black arrows) in L-O2 cells (scale bar 1.0 μm) and the number of autophagosomes per cell was quantified **e**. **f** BECN1 and MAP 1LC3B protein expression levels in L-O2 cells of the indicated groups were analyzed by Western blotting. All results are expressed as the mean ± SD (*P < 0:05; **P < 0:01; ***P < 0.001)

Autophagic flux was then used to further evaluate HucMDE-induced autophagy. Western blot analysis and fluorescent microscopy demonstrated that siRNA-mediated knockdown of ATG5 (Fig. 4a, e, g) or ATG7 (Fig. 4b, e, g), two important genes in the regulation of autophagy, led to decreased HucMDE-induced MAP 1LC3B-II formation and accumulation of MAP 1LC3B puncta in L-O2 cells. We then co-treated L-O2 cells with HucMDEs and autophagic inhibitors (3-MA [10 mM] and Baf [20 nM]), which block the upstream and downstream steps of autophagic flux. Our results showed that 3-MA decreased the HucMDE-induced conversion of MAP 1LC3B-II and accumulation of MAP 1LC3B puncta in L-O2 cells (Fig. 4c, f, h). In contrast, co-treatment of HucMDEs and Baf still led to increased MAP 1LC3B-II formation and accumulation of MAP 1LC3B puncta (Fig. 4d, f, h).

**Fig. 4:** HucMDEs promote autophagic flux in L-O2 cells. **a**, **b** L-O2 cells were transfected with ATG5 or ATG7 siRNAs and were then treated with HucMDEs for 48 h. ATG5, ATG7, and MAP 1LC3B expression levels were examined by Western blotting. **c** L-O2 cells were treated with HucMDEs, 3-MA, or HucMDEs + 3-MA for 48 h. The level of MAP 1LC3B was monitored by Western blotting. **d** L-O2 cells were treated with HucMDEs, Baf, or HucMDEs + Baf for 48 h. The level of MAP 1LC3B was examined by Western blotting. **e** L-O2 cells were transfected with ATG5 or ATG7 siRNAs and were then treated with HucMDEs or DMSO for 48 h, after which they were observed via fluorescent microscopy to evaluate GFP-MAP 1LC3 expression patterns. **f** L-O2 cells were treated with HucMDEs, Baf, or HucMDEs + Baf for 48 h, after which they were observed by fluorescent microscopy to evaluate the GFP-MAP 1LC3 expression patterns. **g**, **h** Percentages of cells with more than four GFP-LC3B dots were quantified of the indicated groups. All results are expressed as the mean ± SD (*P < 0:05; **P < 0:01; ***P < 0.001)

### HucMDEs improve glucose and lipid metabolism by promoting autophagy

We next investigated whether HucMDEs could improve glucose and lipid metabolism in hepatocytes by regulating autophagy. Western blot analysis demonstrated that HucMDEs increased MAP 1LC3B-II formation in PA-treated L-O2 cells, while MAP 1LC3B-II did not increase in response to HucMDEs in PA and 3-MA co-treated L-O2 cells (Fig. 5a). Upregulation of glycolytic enzymes (GCK, PFK, and PK) and p-GSK3β/GSK3β occurred in PA-treated L-O2 cells after HucMDE treatment, while these markers did not increase in response to HucMDEs in PA and 3-MA co-treated L-O2 cells (Fig. 5b, c). Moreover, the expression of hepatic gluconeogenic enzymes (G-6-P and PEPCK) recovered in PA and 3-MA co-treated L-O2 cells after HucMDE treatment (Fig. 5d). PAS staining also demonstrated that HucMDE-induced glycogen accumulation was blocked by 3-MA in PA-treated L-O2 cells (Fig. 5e). Expression of PPARα did not increase in PA and 3-MA co-treated L-O2 cells (despite treatment of HucMDEs) to the levels in PA-treated cells, while downregulation of SREBP-1c expression was partially restored in PA and HucMDEs co-treated L-O2 cells when simultaneously treated with 3-MA (Fig. 5f). These results demonstrate that HucMDEs activate autophagy and, thus, lead to the improvement of glucose and lipid metabolism in PA-treated L-O2 cells.

**Fig. 5:** HucMDEs improve the glucose and lipid metabolism by promoting autophagy. **a** L-O2 cells were treated with PA, PA + HucMDEs, PA + 3-MA, or PA+ HucMDEs + 3-MA. Protein levels of MAP 1LC3B were examined by Western blotting. Glycolysis-related proteins (GCK, PFK, PK) (**b**), glycogen synthesis-related proteins (p-GSK3β, GSK3β) (**c**), and gluconeogenesis-related proteins (G-6-P, PEPCK) (**d**) in L-O2 cells of the indicated groups were detected by Western blotting. **e** PAS staining of L-O2 cells in the indicated groups. **f** SREBP-1c and PPARα in L-O2 cells of the indicated groups were detected by Western blotting. All results are expressed as the mean ± SD (*P < 0:05; **P < 0:01; ***P < 0.001)

### HucMDEs promote autophagy by activating AMPK in L-O2 cells

One of the key molecules that positively regulates autophagy is AMP-activated protein kinase (AMPK) [28]. In addition, our previous research confirmed that AMPK plays an important role in regulating autophagy and metabolism in hepatocytes [23]. We therefore investigated the phosphorylation status of AMPK in T2DM rats and PA-treated L-O2 cells. Western blot analysis showed that HucMDE therapy increased the phosphorylation of AMPK in T2DM rats (Fig. 6a) and PA-treated L-O2 cells (Fig. 6b), which was not seen in the HDEs group. To assess whether HucMDEs induce autophagy through AMPK, AMPK siRNAs were transfected into L-O2 cells. Western blot analysis demonstrated that BECN1 and MAP 1LC3B-II did not increase in AMPK-knockdown L-O2 cells, despite treatment with HucMDEs (Fig. 6c). Moreover, upregulations of BECN1 and MAP 1LC3B-II were restored in L-O2 cells after HucMDE therapy when treated simultaneously with the AMPK inhibitor, Comp C (20 μM; Fig. 6d). In addition, Western blot results demonstrated that HucMDE therapy induced weak increases in glycolytic enzymes (GCK, PFK, and PK) and p-GSK3β/GSK3β levels when treated simultaneously with Comp C relative to these levels in control cells (Fig. 6e, f). Expression of hepatic gluconeogenic enzymes (G-6-P and PEPCK) recovered in PA and Comp C co-treated L-O2 cells after HucMDE treatment (Fig. 6g). PAS staining also demonstrated that HucMDE-induced glycogen accumulation was partially blocked by Comp C in PA-treated L-O2 cells (Fig. 6h). Expression of PPARα increased slightly in PA and Comp C co-treated L-O2 cells, despite the treatment of HucMDEs, to the levels in PA-treated cells. Downregulation of SREBP-1c expression was, however, partially restored in PA and HucMDEs co-treated L-O2 cells when simultaneously treated with Comp C (Fig. 6i). These results further establish that AMPK is a molecular target for HucMDE-induced autophagy.

**Fig. 6:** HucMDEs promote autophagy by activating AMPK in L-O2 cells. Protein levels of p-AMPK and AMPK in the livers (**a**) and L-O2 cells (**b**) of the indicated groups. **c** L-O2 cells were transfected with AMPK siRNA or normal control (NC) siRNA and treated with HucMDEs for 48 h. p-AMPK, AMPK, BECN1, and MAP 1LC3B expression levels were examined by Western blotting. **d** Western blotting analysis of p-AMPK, AMPK, BECN1, and MAP 1LC3B treated with HucMDEs in the absence or presence of Comp C (the AMPK inhibitor, 20 μM) in L-O2 cells. Glycolysis-related proteins GCK, PFK, and PK (**e**); glycogen synthesis-related proteins p-GSK3β and GSK3β (**f**); and gluconeogenesis-related proteins G-6-P and PEPCK (**g**) in L-O2 cells of the indicated groups were detected by Western blotting. **h** PAS staining of the L-O2 cells. **i** SREBP-1c and PPARα in L-O2 cells of the indicated groups were detected by Western blotting. All the results were expressed as mean ± SD (*P < 0:05; **P < 0:01; ***P < 0.001)

## Discussion

The liver plays a major role in maintaining normal blood glucose levels by regulating the balance between the generation and storage of hepatic glucose; however, the ability of the liver in regulating glucose metabolism is impaired in T2DM [29]. With the development of cell-based therapeutic approaches, MSCs have been widely used in the treatment of diabetes, obesity, and liver diseases [30–32]. MSCs can be derived from different sources, such as umbilical cord, bone marrow, adipose tissue, skeletal muscle, liver, lung, and dermal tissues, etc. [33]. Because of the non-invasive acquisition method, no ethical issues, lower immunogenicity, and more stable doubling time, HucMSCs are preferred candidates for cell-based therapies compared to other sources of MSCs [34–36]. In addition, increasing evidence has suggested that exosomes, such as MSCs, show great promise in tissue regeneration and in alleviating T2DM [19]. Therefore, it is important to further elucidate the mechanisms of HucMSCs in improving liver glucose metabolism.

In the present study, we found that HucMDEs decreased fasting blood glucose in T2DM rats, whereas HELFs and HDEs had no beneficial effects. HucMDEs not only improved insulin resistance and increased insulin sensitivity in T2DM rats but also relieved liver dysfunction and improve lipid profiles, as evidenced by significantly decreased serum levels of ALT, AST, TC, and TG. In addition, the expression levels of glycolytic enzymes (GCK, PFK, and PK), p-GSK3β/GSK3β, and lipolytic enzymes (PPARα) were upregulated, whereas hepatic gluconeogenic enzymes (G-6-P and PEPCK) and fatty-acid synthesis enzymes (SREBP-1c) were decreased after HucMDE treatment in T2DM rats and in PA-induced L-O2 cells, indicating that HucMDEs alleviated glucose and lipid metabolism dysfunction both in vivo and in vivo.

Autophagy is a lysosomal degradative process through which misfolded proteins and damaged organelles are sequestered, degraded, and recycled [37]. Previous studies have shown that induction of autophagy in hepatocytes increases insulin sensitivity, suggesting that enhanced autophagy might represent a mechanism for promoting insulin responses and, thus, treating diabetes [38]. However, the effects of MSC-derived exosomes on autophagy in hepatocytes in T2DM remain poorly defined. Our present data showed that autophagy was inhibited in T2DM rats and in PA-induced insulin-resistant cells, while the level of autophagy was elevated after HucMDE intervention. Moreover, liver glucose and lipid metabolism dysfunctions were also improved via HucMDE-enhanced autophagy. These findings indicate that HucMDEs can regulate liver glucose and lipid metabolism in T2DM through inducing autophagy.

The mechanisms that regulate autophagy are complex and have not been fully elucidated. Among the known nutrient-signaling molecules that regulate autophagy, AMPK has been widely demonstrated to be an important intracellular energy sensor functioning on many metabolic stresses and that it achieves energy homeostasis by inhibiting anabolic metabolism and concomitantly activating catabolism [39]. Ren et al. found that AMPK was involved in glycogen synthesis and hepatic gluconeogenesis in a T2DM model [40]. In the present study, we explored the crosstalk between HucMDEs, autophagy, AMPK, and glucose/lipid metabolism in hepatocytes. Our results showed that HucMDE-induced autophagy was disrupted by the AMPK inhibitor, Comp C, or via AMPK knockdown. Furthermore, we demonstrated that introducing inhibition of AMPK reduced the therapeutic effects of HucMDEs on glucose and lipid metabolism dysfunctions. These results indicate that AMPK signaling might be involved in HucMDE-induced autophagy.

## Conclusions

In summary, our present results indicate that HucMDEs effectively alleviated hyperglycemia by improving islet function, promoting glycolysis/glycogen synthesis, and inhibiting gluconeogenesis in T2DM models both in vivo and in vitro and that these efficacies were associated with the upregulation of AMPK-dependent autophagy (Fig. 7). Taken together, our findings elucidate novel molecular mechanisms related to HucMDE-based therapies for preventing and/or treating diabetes and its associated metabolic syndromes.

**Fig. 7:** Working model of HucMDEs in improving hepatic glucose and lipid metabolism. Mesenchymal stem cell-derived exosomes alleviate T2DM by improving the hepatic glucose and lipid metabolism via activating AMPK-dependent autophagy

## Supplementary information

**Additional file 1: Supplementary Figure 1.** Characterization of HucMSCs and uptake of HucMDEs by L-O2 cells. (A) Oil Red O staining of cultured adipogenic HucMSCs. Scale bar: 50 μm. (B) Alizarin red staining of cultured osteogenic HucMSCs. Scale bar: 50 μm. (C) Flow cytometry analysis of HucMSCs-related surface markers (CD105 and CD73) and hematopoietic markers (HLA-DR and CD34). (D) For exosomes uptake in vitro, PBS control (left) and PKH67-labeled HucMDEs (right) were co-cultured with L-O2 cells and cytoskeleton were visualized using rhodamine phalloidin after 24 hours. Scale bar: 25 μm. **Supplementary Figure 2.** Time point of different treat to animal models.

## Data Availability

The datasets used and analyzed during the current study are available from the corresponding authors on reasonable request.

## Abbreviations

MSCs: Mesenchymal stem cells
HucMSCs: Human umbilical cord mesenchymal stem cells
HucMDEs: Human umbilical cord mesenchymal stem cell-derived exosomes
HDEs: HELF-derived exosomes
T2DM: Type 2 diabetes mellitus
IPGTT: Intraperitoneal glucose tolerance test
IPITT: Intraperitoneal insulin tolerance test
AUC: Area under the curve
FBS: Fetal bovine serum
PBS: Phosphate-buffered saline
HFD: High-fat diet
NC: Negative control
TEM: Transmission electron microscopy
ALT: Alanine aminotransferase
AST: Aspartate aminotransferase
MAP 1LC3B: Microtubule-associated protein 1 light chain 3 beta
ATGs: Autophagy-related genes
AMPK: AMP-activated protein kinase
p-AMPK: Phosphorylated AMP-activated protein kinase
